The article "Relationship between Potential Trace Elements Contamination in Sediment and Macrofauna in the Upper Gulf of Thailand" was published in 2023. Journal: J Environ Public Health.

# Relationship between Potential Trace Elements Contamination in Sediment and Macrofauna in the Upper Gulf of Thailand

**DOI:** 10.1155/2023/4231930

**Published:** 2023-01-31

**Authors:** Patarapong Kroeksakul, Arin Ngamniyom, Kun Silprasit, Pakjirat Singhaboot

**Affiliations:** ^1^Faculty of Environmental Culture and Ecotourism, Srinakharinwirot University, Bangkok 10110, Thailand; ^2^Faculty of Agricultural Product Innovation and Technology, Srinakharinwirot University, Nakhon Nayok, Bangkok 26120, Thailand

## Abstract

The relationship between heavy metal contamination in sediment and macrofauna in the upper Gulf of Thailand is presented as an indication of the environmental quality of coastal waters. This study aims to monitor five heavy metal elements (As, Cd, Mn, Ni, and Pb) between sediment and the sandworm (*Perinereis quatrefagesi* (*P. quatrefagesi*)). The geoaccumulation index (*I*_geo_), enrichment factor (EF), and contamination factor (CF), including the pollution load index (PLI), were used for statistical analyses by one-way analysis of variance (ANOVA), and differences in the data were compared using the least significant difference (LSD) test. The sediment heavy metal concentrations were found to decrease (Al > Mn > Pb > Ni > Cd > As), and the quantity of heavy metal contamination in the sediment was not over the emergency point defined by the Pollution Control Department in Thailand. The Mn at the SH and SP points has *I*_geo_ > 0 but <1 and is considered not polluted to moderately polluted. The EF overall is <2 and is deficient in mineral enrichment. The CF of the Samut Sakhon (SH) and Samut Prakan (SP) sites had high Al and Mn values, indicating a low pollution level, but the PLI had an all-site average of 0.0215 ± 0.0252, which is <1. This indicates that the present areas are close to ideal and not polluted. To measure heavy metals in macrofauna, *P. quatrefagesi* was assessed, and concentrations were found to decrease (Mn > Ni > Cd > Pb > As). The Mn between sediment and the sandworm was directly correlated (*r* = 0.976; *p* < 0.01). The sandworm performs as a bioindicator for the quality of coastal sediment, specifically with Mn; thus, the result present at a baseline level may grow in the future if there is no control measure for defensive measures.

## 1. Introduction

Since the upper Thai Gulf connects to the central and eastern regions of Thailand, it has become a hub for industry and agriculture. However, the Thai Gulf is a semienclosed topical sea and serves as a boundary to Malaysia, Cambodia, and Vietnam [1]. The upper zone of the Thai Gulf is connected to the industrial zone and major city and has similar characteristics to ก (Kor Kai is the 1^st^ Thai alphabet). Effectively, locals refer to this zone as “Auw Kor Kai” or “Kor Kai Bay,” and its area encompasses seven provinces: Samut Sakhon, Samut Prakan, Samut Songkhram, Chachoengsao, Chonburi, and Rayong. The major rivers of Thailand that empty into the upper Thai Gulf are the Chao Phraya, Mae Klong, Tha Chin, and Bang Pakong. However, the sandy beaches around the country's tropical regions encourage rapid urban development and tourism. The upper zone of the Thai Gulf also has sandy beaches in the provinces of Chonburi, Rayong, and Phetchaburi and supported over 28 million visitors in 2016 [2, 3]. The sediment comprises the physical dynamics that accommodate and are used by biota, and it serves as a bioindicator of environmental quality [4]. The primary principle of sustainable development is the protection of the environment from human activity, especially in developing countries [5], and one component of protecting the environment is monitoring environmental quality [6]. However, elemental contamination in sediment can also be a secondary source of water quality issues, such as environmental change, and determining the level of heavy metal contamination in sediment is a crucial component of risk evaluation and monitoring in aquatic environments. In the study, we used the geoaccumulation index (*I*_geo_) and enrichment factor (EF) to measure the level of anthropogenic contaminant deposition in sediment and the pollution load index (PLI) to determine the pollutant's concentration in each individual sediment particle.

Macrofauna is an animal group ranging in size from 0.5 to 5 cm that inhabits soft sediment, sand, and mud, and they are associated with fragmentation and decomposition of organic matter as well as nutrient uptake from organic matter, which promotes growth and biofiltration [7, 8]. Furthermore, macrofauna is among the most suitable organisms for bioindicators and bioaccumulators in environmental monitoring studies as they use nutrients from the beach for maintenance and survival [9, 10]. These nutrients act as specific and appropriate biotic tools that can be used when monitoring environmental changes caused by toxic contamination in an area [11, 12], especially for heavy elements that chronically contaminate the food chain. Nevertheless, this study investigates the macrofauna in the sediment of the upper Thai Gulf to assess whether its ratios of heavy metal absorption reflect those of the environment, and the aim is to evaluate the relationship of heavy metal contamination between the beach sediment and macrofauna of the upper zone of the Thai Gulf. This research selected its environmental monitoring areas using literature reporting environmental contamination in the upper zone of the Gulf of Thailand and focused its survey on five heavy metals (As, Cd, Mn, Ni, and Pb) in the sediment and macrofauna. The macrofauna used in this research was the sandworm *Perinereis quatrefagesi* (*P. quatrefagesi*), which is distributed in the sediment around the upper Thai Gulf. *P. quatrefagesi* is responsible for the decomposition of aquatic animals on the coast, which makes it extremely appropriate for indicating the environmental quality [13–15] of the upper zone of the Thai Gulf. This article's presence aims to focus on monitoring elemental contamination in the upper zone of the Thai Gulf area, where there are industrial and agricultural zones with high vulnerability to pollution distribution in the environment, as well as the upper zone of the Thai Gulf being very important to the country's local fishery. The findings of this study suggest that environmental monitoring of sources of pollution will support the continuation of environmental protection policies in the future.

## 2. Methodology

### 2.1. The Sample Collection Areas

After 1958, Thailand developed from an agricultural country to an industrial one by opening the public sector and investing in the country. From 1986−1991, the country developed the industrial sector so quickly that Thailand was designated as a newly industrialized country (NIC) of Asia [16]. Presently, the industrial and service sectors represent the majority of the gross domestic product (GDP) of the country [17]. Concurrently, rural areas are being urbanized, which increasingly affects residential areas in the economic zones, and the populations of high-density cities are growing, which is characteristic of urbanization in the country [18]. The sediment may contain some elemental residue, affecting pollutant levels in the environment.

The sediments around the upper zone of the Thai Gulf have collected during the day from 10 : 00 AM to 3 : 00 PM during an ebbing tide from January to March 2022. The collection points and their distribution in the sample site are Phetchaburi (PB) coordinates Lat 13.224112 Long 99.993748; Samut Songkhram (SS) coordinate Lat 13.361663 Long 100.022530; Samut Sakhon (SH) coordinate Lat 13.586446 Long 100.582095; Samut Prakan (SP) coordinate Lat 13.487892 Long 100.814985; and Chachoengsao (CH) coordinate Lat 13.469204 Long 100.979118, as shown in Figure 1. A quadrate was used to create a margin area on the floor and collect sediment at a depth of 0–5 cm, or about 100–200 g, in the red graphic of the quadrate. However, the sample shall have a weight of about 1.3 kilograms per station and be a homogeneous mixture prior to collection in a polypropylene bag.

### 2.2. Sediment and Macrofauna Collection and Extraction

The sediment was collected from the same sample collection points and mixed homogeneously. Sediment samples weighed approximately 5 kg at each site. The microfauna sample collection was conducted within 0.04 m^2^ of the quadrat sampler at depths of 0–5 cm using mattock plastic. Twenty samples were collected at each site to ensure the collection of *P. quatrefagesi*, and samples were soaked and stored in absolute ethanol before analysis in laboratories. However, successful sample collection of microfauna only occurred at three sites in this study: SH, CH, and SP.

The sediment samples were dried in a hot air oven at 105°C for 168 h until dry. They were then ground using a mortar and pestle. Net no 20 sifted soil was selected for extraction and used in ICP-OES analysis. For this, 2 g of each soil sample was mixed with concentrated hydrofluoric acid (HF), concentrated perchloric acid (HClO_4_), and concentrated nitric acid (HNO_3_) at a 1 : 1 : 1 ratio, totaling 20 mL. Extractions occurred at 500°C in a SpeedDigester K-425 BUCHI (Switzerland) until dry. Each residue was rinsed with 1% HNO_3_ and sieved through filter paper. The supernatant was transferred to a 50 mL volumetric flask, and 1% HNO_3_ was added for continued inductively coupled plasma (ICP) analysis in a PlasmaQuant 9100 series (Germany).

For the sandworm heavy metal analysis, 1 g of wet weight was soaked in 10 mL of concentrated HNO_3_ in a beaker for 24 h. After initial digestion, concentrated HF, HClO_4_, and HNO_3_ were added in a 1 : 1 : 1 ratio, totaling 10 mL. Extractions were performed at 500°C in a SpeedDigester K-425 BUCHI (Switzerland) until dry. Each residue was rinsed with 1% HNO_3_ and sieved through filter paper. The supernatant was transferred to a 20 mL volumetric flask, and 1% HNO_3_ was added for ICP analysis in a PlasmaQuant 9100 series (Germany), and the sample was compared with the ICP multielement standard solution of the AccuStandard (USA).

### 2.3. Geoaccumulation Index (*I*_geo_), Enrichment Factor (EF), and Contamination Factor (CF)

The geoaccumulation index (*I*_geo_) was originally formulated by Muller [19] and is a quantitative measure of pollution in aquatic sediment [20]. It was developed through an understanding of the lithogenic effect. *I*_geo_ was derived using the following formula:

(1) $$\begin{array}{c} I_{geo}=\log\;2\left[\frac{C_{n}}{1.5B_{n}}\right]\text{,} \end{array}$$

where *C*_*n*_ is the measured concentration of an element in the sediment and *B*_*n*_ is the background value of the element. The interpreted values of *I*_geo_ are <0 = not polluted, 0-1 = not polluted to moderately polluted, 1-2 = moderately polluted, 2-3 = moderately to strongly polluted, 3-4 = strongly polluted, 4-5 = strongly to extremely polluted, and >5 = extremely polluted.

The enrichment factor (EF) was derived by the following formula:

(2) $$\begin{array}{c} EF=\left(\frac{C}{RE}\right)\frac{sample}{\left(C/RE\right)background}\text{,} \end{array}$$

where (*C*/RE) sample is the concentration (*C*) of an element to a reference element (RE) in the samples, and (C/RE) background is the concentration (*C*) of an element to a reference element (RE) present in the background. Aluminum (Al) was used as the reference element, as it is a major component of clay, and the interpreted values of EF are <2 = deficiency to mineral enrichment, 2−5 = moderate enrichment, 5−20 = significant enrichment, 20−40 = very high enrichment, and >40=extremely high enrichment.

The concentration factor (CF) is approximated as the ratio of the observed concentration of an element in the sample (*C*_*i*_) to the background level of the same element (*Cb*). The concentration factors were calculated as follows:

(3) $$\begin{array}{c} CF=\frac{Ci}{Cb}\text{.} \end{array}$$

The interpreted values of CF are <1 = low pollution level, 1−3 = moderate pollution level, 3−6 = considerable pollution level, and >6 = very high pollution level.

The background element values for the *I*_geo_, EF, and CF calculations were formulated from the references for As and Ni [21], Al and Pb [22], Cd [23], and Mn [24].

After calculating the concentration factors, they were used to calculate the pollution load index (PLI), which demonstrates the general contamination level [25]. The formula for PLI is as follows:

(4) $$\begin{array}{c} PLI=\sqrt[{n}]{CF1}\;x\;CF_{2}\;x\;CF_{3}\ldots .\;CF_{n}\text{,} \end{array}$$

where CF is the contamination factor of the elements and *n* is the number of observed elements. The interpreted values of PLI are 0 = perfection, <1 = baseline level, and >1 = polluted.

### 2.4. Statistical Analysis

Data were analyzed using a one-way analysis of variance (ANOVA), and the differences in the datasets were compared using the least significant difference (LSD) test with a *p* value of <0.05. Correlations of data were assessed using Pearson's *r* correlation coefficient (*p* < 0.05). All analyses were conducted using Statistical Package for the Social Science (SPSS) v.22.

## 3. Results and Discussion

### 3.1. The Quantity of Heavy Metals in the Sediment of the Thai Gulf

The heavy metal content in the sediment of the upper Thai Gulf was mainly composed of Al, and the average concentration of Al in the samples was 15,642 ± 2,020 mg/kg dry weight. The heavy metal concentrations of the samples exhibited the following pattern: Al > Mn > Pb > Ni > Cd > As. The sediment concentrations of heavy metals in the upper Thai Gulf are presented in Table 1. The concentration of Al was higher at SH (55,358 ± 802 mg/kg) and SP (12,337 ± 770 mg/kg), but not significantly higher at all the sample collection sites. The average sediment As concentration was 0.0612 ± 0.0225, and the As concentration was significantly higher at the PB site than at the SS collection site (*p* < 0.05). The Pb concentrations at the SH, CH, and SP collection sites were not significantly different but were significantly higher than those at the PB and SS sites (*p* < 0.05). The Cd concentration was high at the SP site and significantly different (*p* < 0.05) from the SH, CH, and PB collection sites. The Mn and Ni concentrations were significantly higher at the SP site (*p* < 0.05) than at the SH, CH, PB, and SS collection sites. The concentrations of heavy metals in the sediment of the upper Thai Gulf stand were compared to the emergency points of contamination. In using the scale of land use for agriculture and residential areas by the Pollution Control Department [26], reported metal concentrations are Cd < 67 mg/kg, Mn < 1.7 g/kg, Ni 140.4 mg/kg, Pb < 400 mg/kg, and As < 3.9 mg/kg. Thus, the averages of heavy metals in this series do not exceed the standard for any element. The amount of Al between study sites, however, is not statistically significant, but there are differences in the volume because the nature of the sediment component varies depending on the site. For example, the PB and SS sites have a majority of sand components, whereas the SH, CH, and SP sites almost exclusively have alluvial soil components, which has an impact on the number of elements in the area.

### 3.2. The *I*_geo_, EF, and CF in Sediment of the Upper Gulf of Thailand

The values of *I*_geo_ of the upper Thai Gulf were almost not over 0 (unpolluted) and are presented in Table 2, which aligns with Thongra-ar et al. [27], who presented the geoaccumulation indices (*I*_geo_) of Cd and Ni at values below 0. However, in this study, Mn in the SH and SP collection sites had high *I*_geo_ values over 0 but <1 (0.1873 and 0.5936, respectively). This indicates that SH and SP are not polluted or moderately polluted with Mn. The Al at SH was 0.6376 ± 0.0062, which means that the area was not polluted to moderately polluted with AL. The *I*_geo_ of Al at SH was significantly different (*p* < 0.05) from those at the CH, SP, PB, and SS sites. The *I*_geo_ of As showed no significant differences among any study sites. Mn and Ni *I*_geo_ values showed significant differences among all study sites (*p* < 0.05). Pb *I*_geo_ values between the PB and SS sites were not significantly different, but the two sites were significantly different (*p* < 0.05) from the SH, CH, and SP sites. Nevertheless, the *I*_geo_ of the sediment of the Thai Gulf indicates that the area is mostly not polluted, and some areas are experiencing light to moderate contamination [28].

The EF values in the upper Thai Gulf area are lower than 2, meaning that the sediment has a deficiency in mineral enrichment (Table 2). The EFs of As, Pb, and Cd between the PB and SS sites were not significantly different, but the EFs of As, Pb, and Cd at the PB and SS sites were significantly different (*p* < 0.05) compared to those at the SH, CH, and SP sites. The EF of Mn at the SS site was significantly higher (*p* < 0.05) than that at all other study sites. The EF of Ni at the SS site was significantly higher (*p* < 0.05) than that at the SH, CH, and SP sites but was not significantly different from that at the PB site. The EF values of the upper Gulf of Thailand indicate low coastal heavy metal contamination. Two sample sites had CF values >1: Al (6.512 ± 0.0943, considerable pollution) and Mn (1.539 ± 0.0166, moderate pollution) at SH, and Mn (3.923 ± 0.0263, considerable pollution) and Al (1.451 ± 0.0906, moderate pollution) at SP.

The three analyses illustrate the sediment quality of the upper Gulf of Thailand. The SH and SP collection sites present Al and Mn as ranging from high to over-recommended levels to no pollution. Therefore, PLI is important to use when conducting holistic environmental monitoring of coastal areas in the Gulf of Thailand. The average PLI of all sites in this study was 0.0215 ± 0.0252, which is <1, and indicates that the areas are ideal and not polluted [29, 30]. The PLI values of the SH and SP collection sites were significantly different (*p* < 0.05) from all other sites, as shown in Table 3.

### 3.3. *P. quatrefagesi* in Sediment

Macrofauna is used as bioindicators of coastal environments, as they indicate environmental quality. The sandworm *P. quatrefagesi* is a bioindicator of acute pollution conditions for heavy metals [31, 32]. The sandworms in this study were collected from three sites: SH, CH, and SP. The features and characteristics of the sandworms from the study sites are presented in Figure 2. As concentrations were significantly higher in worms from the SP collection site (*p* < 0.05) than in those from the SH and CH sites, the Pb and Cd contamination in the sandworms from the SH and SP collection sites were significantly different (*p* < 0.05) compared to the CH site. The Mn concentrations in the worms were significantly different (SP > SH > CH, *p* < 0.05), and the Ni concentrations in sandworms from all study sites were not significantly different. The sandworm heavy metal concentrations are presented in Table 4. *P. quatrefagesi* is the optimal bioindicator for copper, manganese, lead, and cadmium [33, 34]. The sandworm is the primary way heavy metals are introduced into the food chain, as they efficiently absorb heavy metals from the environment [35, 36].

### 3.4. Correlation between Heavy Metals in Sediment and *P. quatrefagesi*

The correlation between sample location and heavy metals in sediment and sandworms was evaluated using Pearson's *r* correlation coefficient. Positive correlations were detected in the sediment for manganese (*r* = 0.710; *p* < 0.05), lead (*r* = 0.691; *p* < 0.05), and cadmium (*r* = 0.671; *p* < 0.05), and arsenic was positively correlated between sample location and sandworm (*r* = 0.671; *p* < 0.05). Cadmium heavy metal contamination between sediment and the sandworm was significantly positively correlated (*r* = 0.969; *p* < 0.01); similar correlations were also seen with lead and manganese in the sandworm (*r* = 0.993; *p* < 0.01). Lead in the sandworm and manganese in the sediment were significantly positively correlated (*r* = 0.970; *p* < 0.01), and lead in the sandworm and cadmium in the sandworm were also significantly positively correlated (*r* = 0.954; *p* < 0.01). Lead in the sandworm and nickel in the sediment were significantly positively correlated (*r* = 0.916; *p* < 0.01). The correlations of the other components are presented in Table 5.

### 3.5. Factor Analysis of Heavy Metal Components of Macrofauna and Sediment

The factor analysis of the parameters of the 11 components (heavy metals, sediment, and sandworms) was performed using principal component analysis (PCA). The components found that three PCs had an eigenvalue >1 and explained 88.89% of the cumulative variance in the dataset (Table 6). The component of variance was >10%, as shown in PC1 (62.13%) and PC2 (17.23%) (Table 6, Figure 3). The location was the most important contributor, for which the highest factor load was 0.9394. Location was followed by the primary loading factor, cadmium in sediment (0.8449), and in PC2, the three components were lead in sandworms, cadmium in sandworms, and nickel in sediment. In PC3, arsenic in sediment was found to be an important factor. The PC distributions are presented in Figure 3.

### 3.6. Quality of Sediment around the Upper Gulf of Thailand

The results of the PCA found that location affects the level of heavy metals in sediment and macrofauna. This is also demonstrated by the PLI results, which indicate that the locations of this study are close to ideal. This shows that the coast of the upper zone of the Gulf of Thailand has good environmental quality. However, PLI analysis for surveying environmental quality is only one method for monitoring the environment [37], and it is important in long-term coastal environmental assessments and risk evaluations to use other indicators in conjunction with PLI analysis [38, 39]. Furthermore, in this study, the EF of all components and all areas was <2, which indicates a deficiency in mineral enrichment. Additionally, *I*_geo_ and CF signify no Al or Mn pollution, and Al is the major element of this soil, which is readily absorbed by bottom sediments in the form of metastable compounds [40]. Mn is a product of anthropogenic activity and street dust and is an influential indicator of coastal environmental quality [41, 42]. Its existence is an indicator of human activity on land, which affects the quantity and type of heavy metals in sediment [43, 44].

### 3.7. Performance of Sandworms as Bioindicators for Heavy Metals

The PCA and PC2 results showed that Pb and Cd had high loadings in macrofauna (0.9852 and 0.9654) and were important factors for this analysis. The sandworm (*Perinereis* spp.) is the optimal macrofauna to be collected and used to detect Zn, Cu, Pb, and Cd in the sediment [45, 46]. However, in the heavy metal concentration correlation analyses, only Mn was shown to be directly correlated between sediment and macrofauna (*r* = 0.976; *p* < 0.01). Mn concentration in *Perinereis* spp. is indicative of human activity, which may affect sediment and cause chronic or acute pollution conditions [32]. The ability of polystyrene microplastics to contaminate seawater and sediment is also linked to bioaccumulation within *Perinereis* spp. [47].

## 4. Conclusion

The sediment heavy metal concentrations were found to decrease (Al > Mn > Pb > Ni > Cd > As), and the quantity of heavy metal contamination in the sediment was not over the emergency point defined by the Pollution Control Department in Thailand. Mn at the SH and SP collection sites had an *I*_geo_, which is considered not polluted to moderately polluted and represents a gray area where there is the possibility of pollutants increasing to a crisis point if defensive measures are not taken in the future. The EF overall was deficient in mineral enrichment. The CF of the SH and SP sites had high Al and Mn values, indicating a low pollution level, but the PLI had an all-site perfection level. However, Al is a major component of parent soil sediment in the central region, although Mn levels are rising due to intense traffic and transit that includes industrial zones. This indicates that the present areas are close to ideal and not polluted, but the present result at a baseline level may increase in the future if no defensive measures or controls are taken. To measure heavy metals in macrofauna, *P. quatrefagesi* was assessed, and concentrations were found to decrease (Mn > Ni > Cd > Pb > As). The Mn between the sediment and the sandworm was directly correlated. The sandworm contributes as a bioindicator for the quality of coastal sediment, particularly when Mn is present. However, sediment and macrofauna are important instruments for measuring and monitoring the environmental conditions associated with pollution in the estuarine and Gulf of Thailand ecosystems around the upper zone of the Gulf of Thailand.

## Figures and Tables

**Figure 1:** The characteristics and sample collection sites of the upper Thai Gulf.

**Figure 2:** Characteristics of the sandworms from the different study sites.

**Figure 3:** Results of the PCA for heavy metal contamination distributed in the upper gulf of Thailand: (a) the eigenvalues of components in the principal analysis; and (b) the component of PC loading. PC1 is an element group in the blue ring; PC2 is present in the red ring; and PC3 is present in the yellow ring.

**Table 1:** Concentrations of heavy metals in the sediment of the upper Gulf of Thailand.

Element (mg/kg)	Point of samples collected				
	SH	CH	SP	*P*B	SS
Al	55358 ± 802	5479 ± 59.1	12337 ± 770	2169 ± 131	2866 ± 2713
As	0.0578 ± 0.0096^a^	0.0603 ± 0.0439^a^	0.0591 ± 0.0075^a^	0.0869 ± 0.0062^ab^	0.0421 ± 0.0111^ac^
Pb	7.268 ± 0.1810^a^	3.884 ± 0.1264^b^	15.83 ± 1.228^c^	1.260 ± 0.1413^d^	1.192 ± 0.1112^d^
Cd	1.631 ± 0.1042^a^	1.602 ± 0.0253^ac^	1.809 ± 0.0586^b^	1.542 ± 0.0711^a^	1.538 ± 0.0240^bc^
Mn	495 ± 5.346^a^	219 ± 10.3^b^	1263 ± 6.468^c^	9.959 ± 0.1521^d^	1.963 ± 0.1827^d^
Ni	10.81 ± 0.2651^a^	4.476 ± 0.0378^b^	12.71 ± 0.0793^c^	1.780 ± 0.0682^b^	1.622 ± 0.0882^b^

*Note*. ^abcd^ This mean difference is significant at the *p*-value 0.05 level (LSD); Al = aluminum; A = arsenic; Pb = lead; Cd = cadmium; Mn = manganese; Ni = nickle.

**Table 2:** The *I*_geo_, EF, and CF values of heavy metals in the sediment of the upper Gulf of Thailand.

Element	Index	Point of samples collected				
	*I *_geo_	SH	CH	SP	*P*B	SS
Al		0.6376 ± 0.0062^a^	−0.3668 ± 0.0046^b^	−0.0148 ± 0.0271^c^	−0.7697 ± 0.0261^d^	−0.7701 ± 0.3834^d^
As		−2.345 ± 0.0698	−2.476 ± 0.5226	−2.334 ± 0.0575	−2.165 ± 0.0321	−2.489 ± 0.1125
Pb		−0.4629 ± 0.0107^a^	−0.735 ± 0.0140^b^	−0.1256 ± 0.0330^c^	−1.225 ± 0.0476^d^	−1.249 ± 0.0402^d^
Cd		−0.6035 ± 0.0275^a^	−0.6108 ± 0.0068^a^	−0.5582 ± 0.0139^b^	−0.6276 ± 0.0199^a^	−0.6287 ± 0.118^a^
Mn		0.1873 ± 0.0046^a^	−0.1664 ± 0.0202^b^	0.5936 ± 0.0029^c^	−1.509 ± 0.0066^d^	−2.216 ± 0.0407^e^
Ni		−0.4576 ± 0.0106^a^	−0.8404 ± 0.0036^b^	−0.3872 ± 0.0027^c^	−1.241 ± 0.0147^d^	−1.281 ± 0.3894^e^

	EF	SH	CH	SP	PB	SS
As		0.0002 ± 0.0000^a^	0.0023 ± 0.0000^a^	0.0010 ± 0.0000^a^	0.0058 ± 0.0003^b^	0.0072 ± 0.0044^b^
Pb		0.0003 ± 0.0000^a^	0.0038 ± 0.0000^a^	0.0017 ± 0.0001^a^	0.0097 ± 0.0005^b^	0.0119 ± 0.0073^b^
Cd		0.0000 ± 0.0000^a^	0.0007 ± 0.0000^a^	0.0003 ± 0.0000^a^	0.0020 ± 0.0001^b^	0.0024 ± 0.0015^b^
Mn		0.0058 ± 0.0000^a^	0.0587 ± 0.0006^ab^	0.0261 ± 0.0016^a^	0.1488 ± 0.0088^b^	0.1830 ± 0.1120^c^
Ni		0.0005 ± 0.0000^a^	0.0056 ± 0.0000^ab^	0.0025 ± 0.0001^a^	0.0143 ± 0.0008^bc^	0.0176 ± 0.0107^c^

	CF	SH	CH	SP	PB	SS
Al		6.512 ± 0.0943^a^	0.6445 ± 0.0069^b^	1.451 ± 0.0906^c^	0.2551 ± 0.0154^d^	0.3372 ± 0.3192^d^
As		0.0045 ± 0.0007^a^	0.0047 ± 0.0034^a^	0.0046 ± 0.0005^a^	0.0068 ± 0.0004^ab^	0.0033 ± 0.0008^ac^
Pb		0.3444 ± 0.0085^a^	0.1840 ± 0.0059^b^	0.7503 ± 0.0582^c^	0.0597 ± 0.0066^d^	0.0565 ± 0.0052^d^
Cd		0.3742 ± 0.0238^a^	0.3675 ± 0.0058^a^	0.4149 ± 0.0134^b^	0.3537 ± 0.0163^a^	0.3527 ± 0.0096^a^
Mn		1.539 ± 0.0166^a^	0.6820 ± 0.0321^b^	3.923 ± 0.0263^c^	0.0309 ± 0.0004^d^	0.0060 ± 0.0005^d^
Ni		0.3487 ± 0.0085^a^	0.1444 ± 0.0012^b^	0.4100 ± 0.0025^c^	0.0574 ± 0.0019^d^	0.0523 ± 0.0028^d^

*Note.* ^abcd^ This mean difference is significant at the *p*-value 0.05 level (LSD); *I*_geo_ = geoaccumulation index; EF = enrichment factor; CF = concentration factor; Al = aluminum; As = arsenic; Pb = lead; Cd = cadmium; Mn = manganese; Ni = nickel.

**Table 3:** PLI values of heavy metals in the sediment of the upper Gulf of Thailand.

Area	PLI	Meaning
SH	0.0451 ± 0.0037^a^	Perfection
CH	0.0042 ± 0.0020^b^	Perfection
SP	0.0582 ± 0.0079^c^	Perfection
PB	0.0002 ± 0.0000^b^	Perfection
SS	0.0000 ± 0.0000^b^	Perfection
Average	0.0215 ± 0.0252	Perfection

*Note.* PLI = pollution load index.

**Table 4:** The quantity of heavy metals in sandworms of the upper Gulf of Thailand.

	M-SH	M-CH	M-SP
As	0.00098 ± 0.00005^a^	0.001 ± 0.00009^a^	0.0167 ± 0.0128^b^
Pb	0.0482 ± 0.0139^a^	0.0023 ± 0.00029^b^	0.0413 ± 0.0019^a^
Cd	0.0803 ± 0.0007^a^	0.0238 ± 0.0027^b^	0.0808 ± 0.0067^a^
Mn	14.64 ± 3.395^a^	4.909 ± 0.4838^b^	28.98 ± 0.4070^c^
Ni	0.6716 ± 0.5940	0.1670 ± 0.0912	2.910 ± 4.730

*Note.* ^abc^ This mean difference is significant at the *p*-value 0.05 level (LSD); M = macrofauna (sandworm); As = arsenic; Pb = lead; Cd = cadmium; Mn = manganese; Ni = nickle.

**Table 5:** The correlation between heavy metals in sediment and sandworms.

	Location	S-As	M-As	S-Pb	M-Pb	S-Cd	M-Cd	S-Mn	M-Mn	S-Ni	M-Ni
Location	1										
S-As	0.022	1									
M-As	0.671^*∗*^	−0.039	1								
S-Pb	0.691^*∗*^	−0.007	0.772^*∗*^	1							
M-Pb	−0.134	−0.004	0.307	0.6	1						
S-Cd	0.671^*∗*^	0.064	0.686^*∗*^	0.851^*∗∗*^	0.306	1					
M-Cd	0.007	0.001	0.449	0.724^*∗*^	0.954^*∗∗*^	0.548	1				
S-Mn	0.710^*∗*^	−0.005	0.742^*∗*^	0.993^*∗∗*^	0.58	0.843^*∗∗*^	0.704^*∗*^	1			
M-Mn	0.584	−0.018	0.696^*∗*^	0.970^*∗∗*^	0.648	0.879^*∗∗*^	0.797^*∗*^	0.976^*∗∗*^	1		
S-Ni	0.22	−0.031	0.527	0.850^*∗∗*^	0.916^*∗∗*^	0.635	0.969^*∗∗*^	0.843^*∗∗*^	0.898^*∗∗*^	1	
M-Ni	0.359	0.13	0.612	0.564	0.293	0.567	0.389	0.465	0.445	0.385	1

*Note.* ^*∗*^ = correlation is significant at the 0.05 level (2-tailed); ^*∗∗*^ = correlation is significant at the 0.01 level (2-tailed); S = sediment; M = macrofauna/sandworm; As = arsenic; Pb = lead; Cd = cadmium; Mn = manganese; Ni = nickel.

**Table 6:** The results of PCA of the statistically significant macrofauna and sediment in the upper Thai Gulf.

PCs	Components		
	PC1	PC2	PC3
% of variance	62.13	17.23	9.530
Cumulative %	62.13	79.36	88.89
Eigenvalue	6.83	1.89	1.050
Location	0.9394	−0.1970	−0.0444
S-As	0.0032	−0.0301	0.9597
M-As	0.8268	0.2393	−0.0036
S-Pb	0.8162	0.5623	−0.0112
M-Pb	0.0466	0.9852	0.0308
S-Cd	0.8449	0.3328	0.0815
M-Cd	0.2377	0.9654	0.0413
S-Mn	0.8088	0.5477	−0.0428
M-Mn	0.7331	0.6480	−0.0448
S-Ni	0.4018	0.9115	−0.0269
M-Ni	0.5774	0.2307	0.3433

*Note.* PC = principal component; underlined factor loading is weighted when within 10% of the variation of the absolute value of the highest factor loading in each PC; S = sediment; M = macrofauna.

## Data Availability

All the data generated and analyzed during the current study are included in this published article and are available from the corresponding author upon request.
